The article "City vs. Town residents’ place attachment, perceptions and support for tourism development in a linear World Cultural Heritage Site" was published in 2021. Journal: PLoS One.

# City vs. Town residents’ place attachment, perceptions and support for tourism development in a linear World Cultural Heritage Site

**DOI:** 10.1371/journal.pone.0258365

**Published:** 2021-10-11

**Authors:** Wei Cao, Wendong Yu, Jinhai Xu

**Affiliations:** 1 College of Agriculture, Yangzhou University, Yangzhou, 225009, Jiangsu Province, China; 2 College of Horticulture and Plant Protection, Yangzhou University, Yangzhou, 225009, Jiangsu Province, China; 3 Business School, Yangzhou University, Yangzhou, 225009, Jiangsu Province, China; Universidad de Malaga, SPAIN

## Abstract

This study examines local residents’ place attachment (PA) to the city or town they live and investigates how this attachment influences their perceptions and support for tourism development (ST), as well as comparing the differences of these relationships among the city and town residents in a linear World Heritage Site (WHS) setting. Structural equation model was used to analyze samples of 226 city residents and 235 town residents along the Grand Canal Yangzhou Section, China. The findings suggested that residents’ PA is positively correlated their ST. Results also suggested that the PA-ST effect is partially mediated by residents’ positive perceptions in the city area while fully mediated by residents’ positive and negative perceptions in the town areas. This study could help local governments make heritage development and management policies accordingly for cities and towns along the Grand Canal area.

## 1. Introduction

Human has psychological ties to places, which have been studied and supported by humanistic geographers and environmental psychologists for decades [1]. In the beginning, scholars interpreted this phenomenon through people’s incrementally attaching meaning and experiences to places [2]. Then a series of concepts and models were proposed and developed to further investigate people’s relationship with places, such as place identity [3], place attachment [4,5], sense of place [6], rootedness [7], etc. Thereinto, place attachment has been extensively studied and developed into a multidimensional concept depicting people’s emotional, cognitive, functional, and social connections with places [3,4,8].

The concept of place attachment was initially associated with people’s home environment such as their residences or neighborhoods [1], and then it was adopted in the recreation and tourism related research [9]. Most tourism studies focus on visitors’ place attachment to certain travel destinations [10,11] and how it relates to visitors’ fee spending attitudes [12], site setting perceptions [13], visit motivations [14], place satisfaction [15], place loyalty [16], future visit intentions [17], pro-environment behaviors [15,18], etc. However, most of these study only focused on measuring residents’ place attachment to certain travel destinations, not the entire host living places [19,20]. Studies focusing on the place attachment of local residents in tourist attraction sites are relatively insufficient. Many host places are more than just tourist attractions, they are also well-developed cities or towns with strong historical, cultural, and natural characteristics. It is important to investigate local residents’ place attachment to their dwellings and understand how this attachment would impact their perceptions and support for tourism development.

The article "City vs. Town residents’ place attachment, perceptions and support for tourism development in a linear World Cultural Heritage Site" was published in 2021. Journal: PLoS One.

Since early 1970s, World Heritage Sites (WHS)’s primary goal has been to identify, preserve and protect cultural treasures and natural areas that have outstanding universal values to humanity throughout the world (whc.unesco.org). Those heritage sites are usually important travel destinations that have unignorable economic, sociocultural and environmental contributions to local community development. Destination planning is complicated due to the number of parties involved and affected in the process [21]. As one of the most important stakeholders, heritage sites’ local residents share the responsibility for preserving the outstanding universal value of the heritage as well as utilizing suitable tourism management to achieve sustainable development (whc.unesco.org/en/tourism).

Linear cultural heritages are linear geographically which have “a start and end point, a considerable length and limited width”, such as canals and roads. This type of world heritages, usually passing through multiple administrative and geographical regions, exert extensive and far-reaching influences on the surrounding areas. Since the development of the economy, socio-culture and environment are at different levels along the route, the impacts of the linear heritage tourism on different local communities are most likely to be diversified. Former study compared residents’ responses to tourism development between a rural and a urban heritage sites, but the sites were irrelevant with different characteristics and contexts although within the same nation [22]. Comparative studies of local residents’ responses to heritage tourism upon the same WHS across urban(city) and rural (town) areas are still a paucity.

As one of the most wondrous and magnificent construction in ancient China, the Grand Canal was listed on the UNESCO’s world heritage list in 2014 with 27 sections and 58 heritage sites. Built section by section in different regions and dynasties, connected and expanded to form river systems in Sui Dynasty, and maintained and managed by successive dynasties, the Grand Canal served as a major north-south transportation hub for ancient China with profound political, economic, and cultural influences till today. Entering modern society, the prosperity of the canal has passed, but the protection, management, and sustainable tourism development along the route are ongoing. This research attempts to investigate Yangzhou Grand Canal local residents’ place attachment to the host city or town and how it influences their responses towards heritage tourism development across different regions. By seeing people’s attachment to their place of long-term residence as an essential and intrinsic key factor, this paper aims to discover how residents’ place attachment shape their supportive attitude for tourism which could potentially be mediated by their perceptions, and to compare these effects between city and town residents along the same heritage route.

The article "City vs. Town residents’ place attachment, perceptions and support for tourism development in a linear World Cultural Heritage Site" was published in 2021. Journal: PLoS One.

This study firstly reviews the current literature of place attachment and its subdimensions, residents’ negative and positive perceptions of tourism impact as well as their support for tourism development, subsequently with the proposed hypotheses and conceptual model. Second, the sociodemographic characteristics of respondents are introduced and the research method is described and explained. Finally, the results are widely interpreted, the main findings are discussed and some suggestions are proposed for the future studies.

## 2. Literature review

### 2.1 Place attachment

Place is not just physical space. Its importance has been stressed by scholars as the uniqueness that distinguishes geography from other disciplines. As early as 1970s, humanistic geographer Tuan [2,23] considered space as undifferentiated and it became place only when human got to know it better and endowed it with value, and place was described as the center of meaning constructed by human experience. Relph [24] conserved an intimate conceptual relationship between space and place from a phenomenological point of view, and perceived the specialty of place lies in its ability to spatially organize and centralize individual or group actions, experiences, intentions, and meanings. When people start to attach meaning to a geographical locale, then its physical space becomes place, which could be home, neighborhood, community, city, nation and a variety of places in between [25].

Attachment is the desire to maintain closeness to the object of attachment [26,27]. The mutual relationship and the interdependence of place and people vary in intensity which could be from transitory sensory pleasure to long-lived deeply ingrained attachment [2,25]. People tend to continuously expressing emotions and strengthening connections about particular places [28], and many terms were used to describe the phenomena such as community attachment, place attachment, rootedness and sense of place, among which place attachment was most commonly used for the conceptualization of the affective relationship between people and certain places in literature [4,29,30].

The article "City vs. Town residents’ place attachment, perceptions and support for tourism development in a linear World Cultural Heritage Site" was published in 2021. Journal: PLoS One.

The intensity of attachment may vary at different spatial levels [31,32], such as the house, the street, the neighborhood, the city and the region. Early studies focuses more on the neighborhood or community level which was considered to potentially get more positive results [5,33], then Altman and Low [4] investigated people’s attachment to place at the level of the house, children’s playgrounds, the square, the forest, etc. with one study conducted at three different levels simultaneously [33]. Lately, scholars especially in the field of tourism, broadened their spatial scopes to the national parks and recreation areas [10,18], the national trail [11,13], the regions [34,35], the cities or towns [19,36], etc.

### 2.2 Dimensions of place attachment

Place attachment is a complex and multidimensional concept which deserves systematic analysis [4]. Williams and Roggenbuck [37] initially developed a place attachment scale containing place identity (PI) and place dependence (PD), which had been verified as reliable and valid measures by several authors for different research purposes across different settings [10,12,38]. Proshansky [3] conceptualized PI as the cognitive connection between the self and the physical settings. PI is a concept that has very symbolic and emotional implications since people may attach very personal and abstract meanings to places. While PD is a more concrete concept which mainly refers to individuals’ physical and functional reliance on the living conditions, services and amenities, recreation opportunities or anything supports people’s behavioral goals provided by a place more than an alternative [8,39]. PD conceptually represents the conative domain and embodies the actions or behavioral tendencies of an individual regarding a place [40]. People can be attached to a place because it meets their spiritual or functional needs or both [41], and PI and PD are the two positively and moderately correlated subdimensions under the concept of place attachment [10].

People have tendency to extend their emotional bond with the surroundings to meet their needs [24], and it is the emotions that link all human experiences together [23], so the physical settings gain meanings via the continuous enhancement of people’s emotions. Jorgensen and Stedman [39] regarded sense of place as an attitudinal concept composed of three components: PA, PI and PD, which reflected affect, cognition and conative elements, respectively. The affective component PA stands for sentimental reactions or activities from the sympathetic nervous system which can be revealed by being objectively measured such as heart rate or being subjectively reported by oneself through verbal communications [39]. In order to quantitively measure the affective component, Jorgensen and Stedman [39] adapted some items of PI from Williams and Roggenbuck’s scale and discovered the highest mean scores of this dimension over PI and PD among vacation home owners. Adapted from Jorgenson and Stedman’s conceptualization, Kyle, Mowen [14] incorporated the affective component as a separate subdimension to the concept of place attachment and termed it as affective attachment. They derived measuring items from Williams and Roggenbuck [37]’s scale of PI and proved their reliability and validity. Later researches termed this subdimension as place affect (PAF) and provided sufficient empirical support for its distinction and significance in reflecting the emotional ties between people and place [18,20,36,42,43].

The article "City vs. Town residents’ place attachment, perceptions and support for tourism development in a linear World Cultural Heritage Site" was published in 2021. Journal: PLoS One.

Places often possess strong social attributes since they are often the repositories or contexts where social interactions take place, and people are attached to these social relationships which contribute to people’s interpersonal relationships and “group belonging”, [44,45]. Staying close with neighbors, participating in social activities and having security sense are the main social factors of place attachment [46]. The term “community attachment” is also used to emphasized the role of community when conceptualizing place attachment [47–50]. Mesch and Manor [51] discovered that residents’ connections to their neighborhood were influenced by the level of their social investments within the neighborhood. Hidalgo and Hernández [32] identified that social attachments were stronger than physical attachments in the spatial ranges of houses, neighborhoods, and cities. Although scholars have noticed the existence of the social component, it has not received enough attention in the early place attachment study. Kyle, Mowen [14] added a social dimension termed as social bonding (SB) in their conceptualization of place attachment, which were perceived as another conative component other than PD. Empirical evidences have been found in recreational settings supporting that the provision of social ties by places may lead to higher level of attachment [11,14–16,52]. SB was also a significant predictor of people’s place attachment empirically in built-environment such as residential communities [36,53,54].

The article "City vs. Town residents’ place attachment, perceptions and support for tourism development in a linear World Cultural Heritage Site" was published in 2021. Journal: PLoS One.

Reporting results of the dimensionality of place attachment vary depending on the research contexts in previous study. PI and PD are most commonly recognized and widely-used dimensions which have received consistent empirical support of their reliability and validity in different research contexts. PAF and SB were initially added and confirmed by Kyle, Mowen [14] when studying the relationship between place attachment and place motivation in a US urban park. Rather than constructing a first-order four factor correlated measurement model like Kyle, Mowen [14] did, Brocato [42] built a second-order model with place attachment being the overarching concept and PI, PD, PAF and SB being the four first-order factors. Then he compared it with Kyle’s correlated model with the conclusion that both models provide valid structures for place attachment with identical indices. Although Brocato [42] retained the four factor correlated model based on his theoretical framework, other researchers prefer to use the second-order model and offered empirical support for it, such as studies on the relationship between people’s place attachment, place satisfaction and their pro-environmental behaviors in a natural park context [15,52,55], investigation of the relationship between place attachment, residential satisfaction and community participation in new residential communities [36,53], and research of place attachment’s influence on civic involvements and place loyalty in a new human settlement [54].

There are also scholars only add PAF [17,20,43] or SB [11,16] as the third dimension to construct a first-order correlated measurement. Specifically, in a WHS setting, Hoang, Brown [20] compared the first-order three factor correlated model with the second-order three-dimensional model and received a similar result to Brocato [42] that these two models had identical indices, and Hoang preferred the second-order model for its superiority in parsimony and a better reflection of the complicated definition of place attachment. A second-order four-dimensional structure is used in this study, and place attachment is defined as a second-order concept overarching four first-order factors: PI, PD, PAF and SB, in order to test the suitableness of a more comprehensive measurement of place attachment in a WHS setting while keep the overall model parsimonious.

### 2.3 Residents’ perceptions and support for tourism development

Tourism development generates economic, sociocultural and environmental influences for host places to greater or lesser extents [56]. Local residents’ perceptions are their recognition and awareness to interpret situations and problems of tourism development [57], which can be positive or negative. Economically, a burgeoning tourism industry allows local residents to have increased salary and employment opportunities, but they can also encounter some bad situations such as increased living costs and property prices [58,59]. Socially, local residents can enjoy the improvement in the quantity and quality of recreation and leisure facilities available and the increasing opportunities of demonstrating the traditional arts and cultural identity to a broader audience [58,60], but as the visitor number increases, the traffic and safety may become serious problems [59,61]. Environmentally, a booming tourism industry may increase air and water pollution, produce more waste, disrupt local ecosystems or damage the natural landmarks [62].

The article "City vs. Town residents’ place attachment, perceptions and support for tourism development in a linear World Cultural Heritage Site" was published in 2021. Journal: PLoS One.

Social Exchange Theory (SET) is dominantly utilized when studying residents’ perceptions and the corresponding effects on their attitudes. SET in general is to understand social process based on the exchange of resources between individuals and groups [63]. SET was first brought into tourism studies to elucidate residents’ perception of tourism development by Ap [64], and it suggested that local residents’ perceptions towards tourism were positive when the resource exchange between residents and tourism was high and balanced or unbalanced but high for the residents. Nonetheless, SET is not perfect as it heavily focuses on the economic benefits [65]. The upgraded application of SET emphasizes the interpersonal exchange and holds the view that residents’ values and beliefs play decisive roles of their perceptions of tourism benefits and costs [50,66]. Within this theoretical frame work, factors like residents’ community attachment and environmental attitudes were brought into the study of potential influencing factors contributing to residents’ perceptions of tourism [48–50]. Among these factors, community attachment, a partial concept of place attachment (the socio-cultural dimension of place, Trentelman [9]), was proved to have significant effects on residents’ perceptions in the rural and urban WHS settings [50,66,67].

Social Judgement Theory provides a framework for understanding how people’s prior attitudes influence their perceptions of new stimuli [68]. Kyle, Graefe [13] perceived place attachment as an attitude and the destination’s setting conditions as the stimuli, and discovered that respondents’ level of PI and PD have different impacts on their appraisals and preferences in a natural context. Vong [19] verified the existence of a causal relationship between respondents’ place attachment and perceptions of heritage tourism with PI as the mediating role. However, researches explored the influence of residents’ place attachment on their perceptions is scant. On the basis of the preceding discussions, this research regards place attachment as local residents’ intrinsic nature and could potentially influence their perceptions of tourism development, and then hypothesizes that (Fig 1):

**H1:** Residents’ PA has positive effect on their positive perceptions (PP) of tourism development.
  **H1a:** City residents’ PA has positive effect on their PP of tourism development.
  **H1b:** Town residents’ PA has positive effect on their PP of tourism development.
**H2:** Residents’ PA has negative effect on their negative perceptions (NP) of tourism development.
  **H2a:** City residents’ PA has negative effect on their NP of tourism development.
  **H2b:** Town residents’ PA has negative effect on their NP of tourism development.

The article "City vs. Town residents’ place attachment, perceptions and support for tourism development in a linear World Cultural Heritage Site" was published in 2021. Journal: PLoS One.

**Fig 1:** Proposed model.

The definition of attitudes are people’s response to external events, objects, or incentives [69]. Local residents generally hold supportive, opposing or neutral attitudes towards tourism development. The success and sustainability of tourism development is inseparable from local residents’ supportive attitude [70]. Residents’ PP and NP of tourism impacts are crucial indicators of their support for tourism development [48,49,71]. Several scholars applied SET and identified that when residents perceived benefits from tourism development outweigh the cost, they would show supportive attitude [48,50]. On the contrary, residents decreased their supporting for future tourism development if they perceived more negative impacts than the positive [72]. Sirivongs and Tsuchiya [57] proved that positive perceptions of local residents had strong impact on their attitudes while negative perceptions showed no influence on their attitudes in a national setting. In terms of the rural-urban differences, several studies showed that urban residents perceived more benefits brought by tourism development but were also more concerned of the potential damages, while rural residents in general were less aware of the possible benefits and costs [59,60]. Rasoolimanesh, Ringle [22] discovered that residents’ perceptions in rural and urban WHS settings have significant different effects on support for tourism. Based on the discussions above, we propose that (Fig 1):

**H3:** Residents’ PP have positive effect on their support for tourism development (ST).
  **H3a:** City residents’ PP have positive effect on their ST.
  **H3b:** Town residents’ PP have positive effect on their ST.
**H4:** Resident’s NP have negative effect on their ST.
  **H4a:** City residents’ NP have negative effect on their ST.
  **H4b:** Town residents’ NP have negative effect on their ST.

The article "City vs. Town residents’ place attachment, perceptions and support for tourism development in a linear World Cultural Heritage Site" was published in 2021. Journal: PLoS One.

The following hypotheses are set up to further examine the direct effect of residents’ PA on their support and the mediating role of their perceptions:

**H5:** Residents’ PA has positive effect on their ST.
  **H5a:** City residents’ PA has positive effect on their ST.
  **H5b:** Town residents’ PA has positive effect on their ST.
**H6:** Residents’ PP play a mediating role between their PA and ST.
  **H6a:** City residents’ PP play a mediating role between their PA and ST.
  **H6b:** Town residents’ PP play a mediating role between their PA and ST.
**H7:** Residents’ NP play a mediating role between their PA and ST.
  **H7a:** City residents’ NP play a mediating role between their PA and ST.
  **H7b:** Town residents’ NP play a mediating role between their PA and ST.

## 3. Methodology

### 3.1 Study area

With a history of over 2500 years, the Grand Canal is a vast waterway system which starts at China’s capital city Beijing in the north and ends in Zhejiang province in the south, passing through two municipalities, six provinces, and 25 prefecture-level cities and linking five of China’s main river basins.

Located at the Jiangsu Plain, Yangzhou Section of the Grand Canal covers a total length of 151.3 kilometers, including six waterways and ten heritage sites along. As one of the oldest and most important section of the Grand Canal, this section played an important role in grain transportation and salt distribution, which contributed to the prosperity of the adjacent cities and towns. Yangzhou is a city that rose and fell with the canal, and now it is a tourist city with rich history and culture that owns the most heritage sites of the Grand Canal. Among the heritage waterways and sites, three waterways (Former Waterway of Hangou Canal, Ancient Canal of Yangzhou, and Guazhou Canal) and six sites (Slender West Lake, Temporary Palace at Tianning Temple, Ge Garden, Wang Lumen’s Residence, Salt Ancestral Temple and Lu Shaoxu’s Residence) are within the downtown urban areas of the city of Yangzhou (which are Guangling District and Hanjiang District), while the rest three waterways (Li Canal, Former Waterway of Gaoyou in Ming and Qing Dynasties, and Former Waterway of Shaobo in Ming and Qing Dynasties) and four sites (Liubao Lock, Yucheng Post, Ancient Shaobo Dike, and Shaobo Docks) belong to the county (town) or rural areas under the prefecture-level city of Yangzhou (which are Jiangsu County, Gaoyou County and Baoying County).

The city area of the Grand Canal Yangzhou Section, composed of Guangling District and Hanjiang District, covers an area of 248 km^2^ with a population of 1.2 million (until April 2018). This area has started its historical preservation and tourism development for over 30 years, taking the development of Slender West Lake Scenic Area as a starting point. With Slender West Lake being a national 5A-rated tourist attraction, there are eleven 4A-rated tourist attractions within the downtown Yangzhou, and half of those attractions are historical sites with rich cultural, historical and artistical values. The town areas of the Grand Canal Yangzhou Section which go through Jiangdu County, Gaoyou County and Baoying County cover an area of 4763 km^2^ with a population of around 2.8 million (until April 2018). Shaobo Town and Yucheng Post were planned and developed for heritage tourism after the Grand Canal was declared a WHS in 2014 and were approved as 4A-rated tourist attractions in recent years, while Liubao Lock is still underdeveloped for tourism. This is a very different situation from downtown Yangzhou where tourism has been developing long before the Grand Canal was listed. This study employs city and town residents around the ten heritage sites for the empirical analysis (Fig 2).

The article "City vs. Town residents’ place attachment, perceptions and support for tourism development in a linear World Cultural Heritage Site" was published in 2021. Journal: PLoS One.

**Fig 2:** Location map of the study area.

### 3.2 Data collection and sample profile

Onsite surveys were conducted from October to December in 2020 by a team of four students for data collection of this study. In order to gain a representative sample, questionnaires were distributed among passers-by near the heritage sites adopting three forms of randomization strategies. One was time selection, which meant team members went to the sites to conduct the survey at random hours throughout the daytime on both weekdays and weekends. The other one was geographical location, which meant team members collected about the same number of samples in each site in the city area (six sites, within 2km of each site) and in the town area (four sites, within 3km of each site), respectively, as well as stationed at different spots within each site at the same intervals. Most city sampling occurred on the streets and squares while most town sampling was done at local public spaces. The last strategy was systematic interception of individuals when they approached the teams. People were asked if they were residents nearby and whether they would like to participate in this survey. A total of 489 (93.5% response rate) residents completed the questionnaires and 461 of them were finally confirmed as valid after screening. A number of 461 samples composed of 226 city samples (48 samples from Slender West Lake, 35 samples from Temporary Palace at Tianning Temple, 45 samples from Ge Garden, 32 samples from Wang Lumen’s Residence, 31 samples from Salt Ancestral Temple and 35 samples from Lu Shaoxu’s Residence) and 235 town samples (61 samples from Liubao Lock, 72 samples from Yucheng Post and 102 samples from Ancient Shaobo Dike and Shaobo Docks) were sufficient for this research.

The article "City vs. Town residents’ place attachment, perceptions and support for tourism development in a linear World Cultural Heritage Site" was published in 2021. Journal: PLoS One.

Table 1 shows the socio-democratic characteristics of the samples. There were more female participants than male, especially in the town group. Respondents varied in different age groups ranging from 18 to more than 60 years old, in which the majority of them were relatively young, especially in the city group (68.6% and 44.3% were between 18 to 39 years old in the city group and the town group, respectively). Respondents from the city group were generally better educated than those from the town group, since more people owned bachelor’s degree or higher. 75.5% of all the participants were native born and bred and the rest settled here for work, marriage, etc. 93.5% of all the survey respondents knew Yangzhou Section of the Grand Canal were a WHS and 82.6% of them were aware that China was promoting the development of Grand Canal National Cultural Parks.

**Table 1:** Profile of respondents.

Characteristics	n	Percentage	n	Percentage	n	Percentage
	Combined group		City group		Town group	
**Gender**						
Male	194	42.1	108	47.8	86	36.6
Female	267	57.9	118	52.2	149	63.4
**Age, years**						
18–29	127	27.5	76	33.6	51	21.7
30–39	132	28.6	79	35.0	53	22.6
40–49	78	16.9	31	13.7	47	20.0
50–59	55	11.9	14	6.2	41	17.4
60 and above	69	15.0	26	11.5	43	18.3
**Marital status**						
Single	95	20.6	58	25.7	37	15.7
Married	354	76.8	166	73.5	188	80.0
Divorced or Widowed	12	2.6	2	0.9	10	4.3
**Education level**						
Primary school or below	35	7.6	1	0.4	34	14.5
Middle school	99	21.5	15	6.6	84	35.7
High school or technical	133	28.9	63	27.9	70	29.8
Undergraduate	185	40.1	139	61.5	46	19.6
Postgraduate	9	2.0	8	3.5	1	0.4
**Identity**						
Yangzhou native born and raised	348	75.5	172	76.1	176	74.9
Immigrant from other regions	113	24.5	54	23.9	59	25.1
**Length of residence (years)**						
0–9	85	18.4	40	17.7	45	19.1
10–19	65	14.1	23	10.2	42	17.9
20–29	88	19.1	61	27.0	27	11.5
30–39	81	17.6	47	20.8	34	14.5
40 and above	142	30.8	55	24.3	87	37.0

### 3.3 Measures

The study examines the relationship between local residents’ PA and ST as well as the mediating role of their perceptions. A questionnaire designed into two sections was utilized as the instrument of the study, one was to collect demographic information and the other was composed of the measuring items of the seven constructs, which were adapted from scholarly references to measure residents’ PA to their living city or town, their perceptions, and support for the tourism development of the Grand Canal. PI and PD were measured using four items respectively developed and validated by Williams and Vaske [10]. PAF was measured by a 4-item scale developed and tested by Jorgensen and Stedman [39] and Hoang, Brown [20]. The three items of SB were adapted from Kyle, Mowen [14] and Hesari, Peysokhan [36]. Measuring items of residents’ perceptions and support for tourism were adapted from Rasoolimanesh, Roldán [66], Rasoolimanesh, Jaafar [67], and Vong [19]. The item list was not meant to be exhaustive as long as it served the research goal well, and the average response time of the participants was three minutes. The questionnaire was answered on a 5-point Likert scale, in while 1 refers to *strongly disagree* and 5 refers to *strongly agree*. A ‘do not know’ option was also provided to the survey participants for their non-attitudes to make sure that the measurement is reliable and valid [73].

The article "City vs. Town residents’ place attachment, perceptions and support for tourism development in a linear World Cultural Heritage Site" was published in 2021. Journal: PLoS One.

### 3.4 Preliminary statistical verification

Before testing the proposed hypotheses, the normality of the data and common methods variance (CMV) were examined for statistical verifications. Each variable’s skewness and kurtosis were checked to see if the data was normally distributed. The results demonstrated that all the skewness and kurtosis were between -1.027 to +1.779, lower than the cutoff of 2 and 7 [74], respectively. Therefore the normality of the distribution of data was sustained, which was the foundation for applying maximum likelihood estimation in SEM [75]. By checking the Mahalanobis distance of all the data samples, six outliers were removed from the data to decrease multivariate kurtosis [76].

The design of the questionnaire and the data collection process were conducted according to Podsakoff, MacKenzie [77] in order to decrease CMV, but CMV was still a potential problem since all the measures were generated using the same instrument by the same respondent [78]. Two statistical analysis were performed to assess the possible existence and severity of CMV. First, Harman’s one-factor test was done on the constructs and subscales in the theoretical model and the test result showed that the most covariance explained by one factor was 35.15%, indicating that CMV was not likely a problem of our results [79]. Second, a single confirmatory factor analysis (CFA) was conducted and results showed that the one common factor model did not fit the data well (CFI = 0.683, RMSEA = 0.129) and the one factor model was significantly worse than the proposed multifactor model through chi-square test (Δχ^2^ = 1649.55, Δ*df* = 21, p<0.001). Both analyses alleviated the CMV concern in this study.

### 3.5 Ethics statement

Ethics approval for the study was given by Yangzhou University, Medical College Ethics Committee (Approval number YXYLL-2020-135). The first author designed the questionnaire independently, and the accuracy, consistency and completeness of all questions in the questionnaire were carefully checked. All the data was collected under the supervision of the first author. Informed consent was obtained in the beginning of the questionnaire, and all the participants were told that the data would be used for research purpose only.

The article "City vs. Town residents’ place attachment, perceptions and support for tourism development in a linear World Cultural Heritage Site" was published in 2021. Journal: PLoS One.

## 4. Results

### 4.1 Measurement model

A two-step SEM procedure of developing the measurement model firstly and evaluating the structural model secondly [80], analyzed by AMOS 24.0, was used to test the research hypothesis. CFA was performed on the combined group (461 samples), the city group (226 samples) and the town group (235 samples) separately with the four first-order subscales of PA and the other three constructs of PP, NP and ST in order to assess whether the measurement model accurately reflect the desired seven constructs based on the maximum likelihood estimation. Item PAF4 was removed from the measurement due to its low squared multiple correlations in all three groups (0.30, 0.32 and 0.31 in the combined, the city and the town group, respectively) where a threshold of 0.36 was recommended by Fornell and Larcker [81], and NP3 was eliminated because of its substantially low squared multiple correlations in the town group (0.15) as well as in the combined group (0.31). Item PI2, PD4 and RP5 were deleted due to their large residual covariance with other items [82] resulting high RMSEA (above 0.08) and high ratio of χ^2^ to degree of freedom (above 3.0). Theoretical considerations were reviewed to make sure that elimination of these items would not influence the conceptual nature of the respective latent constructs nor their subscales.

Descriptive statistics of the variables are shown in Table 2. The mean values for city and town residents’ PA were not statistically different after conducting a t-test (p = 0.43), which indicated that residents of the two groups had similar level of attachment to their city or town. The statistics also showed that the city residents have similar levels of PP, NP and ST with the town residents.

**Table 2:** Descriptive analysis.

Construct & Item		Mean value	Standard deviation	Mean value	Standard deviation	Mean value	Standard deviation
		Combined group		City group		Town group	
**Place Attachment (PA)**							
*Place Identity (PI)*							
PI1	I identify strongly with X.	4.24	.76	4.28	.72	4.20	.80
PI3	X is very special to me.	4.12	.80	4.19	.79	4.06	.80
PI4	X means a lot to me.	4.24	.78	4.31	.76	4.17	.80
*Place Dependence (PD)*							
PD1	X is the best place for me to live.	4.03	.90	4.01	.92	4.06	.89
PD2	I get more satisfaction out of living here than any other place.	3.99	.86	4.00	.89	3.99	.83
PD3	For doing the things that I enjoy most, no other place can compare to X.	3.93	.92	3.92	.97	3.94	.87
*Place Affect (PAF)*							
PAF1	I feel happiest when I’m living here.	4.02	.79	4.06	.77	3.97	.81
PAF2	X is my favorite place to be.	3.95	.89	4.02	.89	3.88	.90
PAF3	I really miss X when I’m away from it for too long.	4.11	.77	4.15	.73	4.08	.80
*Place Social Bonding (SB)*							
SB1	My family/friends would be disappointed if I were to start living in other places.	3.81	.85	3.78	.83	3.83	.88
SB2	Many of my family /friends prefer living here over other places.	3.98	.78	4.03	.70	3.93	.85
SB3	My family and I enjoy the relationships with our neighbors.	4.09	.70	4.04	.70	4.14	.70
**Positive Perceptions (PP)**							
PP1	Tourism development TGC would create more jobs for my community.	3.98	.79	4.04	.74	3.93	.83
PP2	Our standard of living would increase considerably because of tourism development of TGC.	4.11	.76	4.10	.77	4.11	.75
PP3	Tourism development of TGC provides more infrastructure and public facilities like roads, shopping, etc.	4.10	.72	4.04	.76	4.16	.68
PP4	Tourism development of TGC would help the preservation of local culture.	4.24	.65	4.21	.67	4.26	.63
**Negative Perceptions (NP)**							
NP1	Local residents’ daily life would suffer from the tourism development of TGC.	2.94	1.08	3.08	1.09	2.80	1.05
NP2	The construction of hotels and other tourist facilities would destroy the natural environment.	3.01	1.13	3.10	1.22	2.93	1.02
NP4	Tourism development of TGC would cause traffic congestion.	2.61	1.07	2.70	1.11	2.53	1.03
**Support for Tourism Development (ST)**							
ST1	I support tourism development of TGC and would like to see it become an important part of my community.	4.17	.63	4.12	.64	4.22	.61
ST2	Tourism development of TGC should be actively encouraged in my community.	4.23	.65	4.21	.68	4.24	.62
ST3	The government was correct in supporting the promotion of tourism development of TGC.	4.26	.64	4.20	.66	4.31	.61
ST4	It is important to develop plans to manage the conservation of historical sites and the growth of tourism.	4.36	.63	4.42	.60	4.30	.65

Note: X stands for the place each group of respondents reside.

The article "City vs. Town residents’ place attachment, perceptions and support for tourism development in a linear World Cultural Heritage Site" was published in 2021. Journal: PLoS One.

Subsequently, CFA was performed separately on the adjusted second-order PA construct among the three groups to test whether the second-order four-dimension structure of PA was a good replacement of the four first-order factors correlated model in this research context. Table 3 showed that the model fit indices were all at acceptable levels. The calculated target coefficients [83] were 0.92, 0.99, 0.87 for the combined, the city and the town group, respectively, meaning around ninety percent of the variation in the first-order could be explained by the second-order in each group. This provided sufficient support for the implementation of the second-order PA construct in this study.

**Table 3:** Measurement model indices for PA construct.

Group	χ2		Target coefficient	*df*	χ2/*df*	RMSEA	SRMR	CFI	TLI
	1st-order model	2nd-order model		2nd-order model					
Combined Group	102.198	111.047	0.920	50	2.221	0.052	0.030	0.981	0.974
City Group	82.225	82.528	0.996	50	1.651	0.054	0.035	0.976	0.968
Town Group	104.090	119.384	0.872	50	2.388	0.077	0.040	0.963	0.951

The adjusted measurement model (Table 4), comprised of seven latent constructs and 23 observed items, demonstrated a good model fit with a significant χ^2^ of 337.89, 335.46, and 333.79 (*df* = 209, p<0.001) for the three groups respectively which were highly impacted by the large size of sample. The ratio of χ^2^ to the degrees of freedom (χ^2^/*df*) were 1.62, 1.61 and 1.60, which were all lower than the recommended threshold of 3.0 [84]. Another commonly used model indices of the three groups lend credence to the measurement model: all the root mean square errors of approximation (RMSEA) and the standardized root mean square residuals (SRMR) were no more than 0.08, and the comparative fit index (CFI) and the Tucker Lewis index (TLI) were all higher than the cutoff of 0.90 [75].

**Table 4:** Overall measurement model indices.

Group	χ2	*df*	χ2/df	RMSEA	SRMR	CFI	TLI
Combined Group	337.890	209	1.617	0.037	0.033	0.977	0.972
City Group	335.463	209	1.605	0.052	0.050	0.949	0.938
Town Group	333.793	209	1.597	0.051	0.043	0.962	0.954

The reliability of the model, given the composite reliability (CR) scores for each variable in all the three groups, were ranging from 0.67 to 0.90 (Table 5), most of which were greater than the recommended cut-off of 0.70 [75,81] with one exception (0.674 for SB construct of the city group, close to 0.70), indicating that the scales were reliable. Construct validity (including both convergent and discriminant validity) demonstrates to what degree the items of a construct measure what they are supposed to measure [85]. Convergent validity (Table 5) was supported by both statistically significance (p < .001) of all the item loadings ranging from 0.52 to 0.94 [80,86,87]; and average of variance extracted (AVE) values of all constructs (Table 5) were higher than the recommended threshold of 0.50 [75,81] with one exception of 0.41, while greater than 0.36 was acceptable according to Fornell and Larcker [81]. These values provided adequate evidence of convergent validity [75]. Discriminant validity means each construct should be statistically different from one another, requiring all the inter-factor correlation estimates lower than the square roots of the corresponding AVE values [75,81]. Table 6 shows that the square root of each construct’s AVE value exceeded its correlation with other constructs, providing support for discriminant validity [81,88]. For instance, in the combined group, the square root of residents’ PA was 0.816 while its correlation with PP, NP and ST were 0.565, -0.128, 0.491, respectively.

The article "City vs. Town residents’ place attachment, perceptions and support for tourism development in a linear World Cultural Heritage Site" was published in 2021. Journal: PLoS One.

**Table 5:** CFA results for measurement models of constructs.

Construct & Item	Factor loading	CR	AVE	Factor loading	CR	AVE	Factor loading	CR	AVE
	Combined group			City group			Town group		
**Place Attachment (PA)**		.888	.666		.879	.647		.897	.687
*Place Identity (PI)*		.820	.604		.792	.560		.842	.644
PI1	.687			.730			.655		
PI3	.811			.740			.869		
PI4	.826			.773			.865		
*Place Dependence (PD)*		.855	.664		.851	.655		.862	.678
PD1	.804			.837			.767		
PD2	.875			.823			.936		
PD3	.762			.767			.754		
*Place Affect (PAF)*		.848	.651		.814	.595		.876	.702
PAF1	.796			.802			.793		
PAF2	.854			.812			.888		
PAF3	.769			.695			.829		
*Place Social Bonding (SB)*		.747	.500		.674	.414		.807	.589
SB1	.739			.764			.724		
SB2	.795			.626			.934		
SB3	.568			.516			.610		
**Positive Perceptions (PP)**		.824	.545		.817	.534		.835	.563
PP1	.637			.597			.688		
PP2	.891			.899			.878		
PP3	.770			.774			.775		
PP4	.623			.611			.638		
**Negative Perceptions (NP)**		.814	.596		.821	.605		.805	.584
NP1	.850			.828			.880		
NP2	.785			.797			.766		
NP4	.671			.703			.626		
**Support for Tourism Development (ST)**		.843	.574		.817	.531		.873	.633
ST1	.740			.678			.789		
ST2	.822			.876			.788		
ST3	.790			.723			.833		
ST4	.669			.612			.770		

Notes: CR: Composite reliability. AVE: Average variance extracted.

**Table 6:** Discriminant validity matrix.

	Combined group				City group				Town group			
	PA	PP	NP	ST	PA	PP	NP	ST	PA	PP	NP	ST
PA	**.816**				**.804**				**.829**			
PP	.565	**.738**			.487	**.731**			.636	**.750**		
NP	-.128	-.010	**.772**		-.023	.132	**.778**		-.243	-.160	**.764**	
ST	.491	.630	-.162	**.758**	.479	.601	.001	**0.729**	.505	.657	-.329	**.796**

Note: Square root of AVE in bold on diagonals; Off diagonals are Pearson correlation of constructs.

### 4.2 Structural model and multi-group analysis

SEM was employed on the whole data samples, the city sample group and the town sample group, respectively, to examine and analyze the research hypotheses. The proposed second-order structural equation model (Table 7), revealed good fits to all three sample groups. Chi-square adjusted for the degree of freedom (χ^2^/*df*) is 1.74, 1.72 and 1.63, respectively, which are all less than 3.0. The RMSEA and SRMR for the three groups are all less than 0.08; the CFI and TLI are all above 0.90, and most of which are greater than 0.95. All the most commonly used indices confirmed the goodness of model fit of the three groups.

The article "City vs. Town residents’ place attachment, perceptions and support for tourism development in a linear World Cultural Heritage Site" was published in 2021. Journal: PLoS One.

**Table 7:** Structural equation model indices.

Group	χ2	*df*	χ2/df	RMSEA	SRMR	CFI	TLI
Combined Group	384.986	221	1.742	0.040	0.041	0.970	0.966
City Group	379.068	221	1.715	0.056	0.064	0.936	0.927
Town Group	360.613	221	1.632	0.052	0.045	0.957	0.951

Hypothesis testing of structural model results was shown in Table 8 and Fig 3. The direct path coefficient from the second-order predictor (PA) to the criterion variable (ST) was significant in the combined group (Hypothesis H5: β = 0.115, p<0.05), indicating that Yangzhou residents’ PA to their city or town do have a significant positive impact on their ST towards the Grand Canal’s tourism development. However, situations varied in the two sub-regional groups. This direct effect was significantly positive in the city group (Hypothesis H5a: β = 0.225, p<0.01) but not significant in the town group (Hypothesis H5b: β = -0.033, p>0.05).

**Fig 3:** SEM results for the three groups.

**Table 8:** Hypothesis testing of structural model.

	Combined group			City group			Town group			χ^2^ Difference	
Relationships		Std. Est.	t-value		Std. Est.	t-value		Std. Est.	t-value	χ^2^	P
PA —> PP	H1	0.625***	8.845	H1a	0.525***	5.461	H1b	0.724***	7.012	6.176	*
PA —> NP	H2	-0.137*	-2.547	H2a	-0.022	-0.288	H2b	-0.264***	-3.423	5.077	*
PP —> ST	H3	0.659***	8.796	H3a	0.594***	5.669	H3b	0.745***	6.720	.002	ns
NP —> ST	H4	-0.164***	-3.871	H4a	-0.097	-1.534	H4b	-0.233***	-3.843	2.537	ns
PA —> ST	H5	0.115*	1.999	H5a	0.225**	2.839	H5b	-0.033	-.364	4.629	*

Note: * p<0.05,

** p<0.01,

*** p<0.001. ns = not significant.

Relationships between residents’ PA, PP and ST were identical among all three groups. There were significantly positive impacts of residents’ PA on their PP (Hypothesis H1: β = 0.625, p<0.001; H1a: β = 0.525, p<0.001; H1b: β = 0.724, p<0.001) and significantly positive influence of residents’ PP on their ST (Hypothesis H3: β = 0.659; p<0.001; H3a: β = 0.594, p<0.001; H3b: β = 0.745, p<0.001) across all the three groups.

However, relationships associated with residents’ NP were diversified among the three groups. The proposed significantly negative impact of resident’s PA on their NP were supported in the combined group and the town group (Hypothesis H2: β = -0.137, p<0.05; H2b: β = -0.264, p<0.001) but not supported in the city group (Hypothesis H2a: β = -0.022, p>0.05). The effects of residents’ NP on their ST were significantly negative in the combined group and the town group (Hypothesis H4: β = 0.-164, p<0.001; H4b: β = -0.233, p<0.001) but not significant in the city group (Hypothesis H4a: β = -0.097, p>0.05).

The article "City vs. Town residents’ place attachment, perceptions and support for tourism development in a linear World Cultural Heritage Site" was published in 2021. Journal: PLoS One.

The mediating effects of residents’ PP and NP on the association between their PA and ST were further examined. A bootstrap analysis with 95% bias-corrected confidence intervals (CI) and 5000 resamples were used in this study to analyze the mediation effects [89], and the relationship is significant if the CIs does not include zero.

PP significantly mediates the effect of PA on ST in the combined group, the city group and the town group (Hypothesis H6: β = 0.412, Boots CI: [0.309, 0.528]; H6a: β = 0.312, Boots CI: [0.185, 0.469]; H6b: β = 0.539, Boots CI: [0.401, 0.760]), giving support to hypotheses H6, H6a and H6b (Table 9). Nevertheless, the mediation effects of NP on the association between PA and ST was only significant in the combined group and the town group (Hypothesis H7: β = 0.023, Boots CI: [0.005, 0.052]; H7b: β = 0.061, Boots CI: [0.019, 0.129]), but not significant in the city group (H7a: β = 0.002, Boots CI: [-0.013, 0.029]), which only support hypotheses H7 and H7b. The mediation test shows that city residents’ PP partially mediate the relationship between their PA and ST, while town residents’ PP and NP fully mediated this relationship.

**Table 9:** Results of mediation analyses.

	Combined group				City group				Town group			
			bias-corrected 95%				bias-corrected 95%				bias-corrected 95%	
	Std. Est.	S.E.	Lower	Upper	Std. Est.	S.E.	Lower	Upper	Std. Est.	S.E.	Lower	Upper
PA-PP-ST	0.412***	.056	.309	.528	0.312***	.073	.185	.469	0.539***	.088	.401	.760
PA-NP-ST	0.023*	.011	.005	.052	.002	.010	-.013	.029	0.061**	.028	.019	.129
Total indirect effect	0.435***	.057	.330	.554	0.314***	.072	.187	.471	0.601***	.094	.450	.827
Total effect	0.550***	.041	.465	.628	0.539***	.069	.394	.668	0.568***	.051	.465	.663

Note: * p<0.05,

** p<0.01,

*** p<0.001.

Multi-group analysis in SEM was carried out to investigate the effects of the two sub-regional groups concerning in residents’ PA, PP, NP and ST. Adopting the analytical strategy of Singh [90] and Gu, Fan [91], evaluation of whether the path coefficients were different across the city and the town groups was performed. The results are presented in Table 8. It is discovered that the path coefficients, which deal with the impact of PA on PP (p<0.05), PA on NP (p<0.05) and PA on ST (p<0.05), were confirmed to differ significantly between the city and the town group in the Chi-square testing, while differences of the impact of PP on ST and NP on ST between the two groups were not significant.

The article "City vs. Town residents’ place attachment, perceptions and support for tourism development in a linear World Cultural Heritage Site" was published in 2021. Journal: PLoS One.

## 5. Discussions

This study investigated the relationship between local residents’ PA and their ST with the possible mediating roles of residents’ PP and NP in Yangzhou Grand Canal region. The Grand Canal is a socioeconomically and culturally holistic region, but it is spatially and regionally linear passing through multiple provinces and municipalities of China, which could lead to different local residents’ responses of heritage tourism development. Therefore, this study included a comparison between the city residents and the town residents to examine the differences of the proposed relations.

The study confirmed that the four interrelated factors of PI, PD, PAF and SB were reliable and convergent dimensions of measuring local residents’ attachment to a WHS, and the second-order structure of PA were efficient. The findings are in consistent with former studies on national park settings [15,55] and urban residential settings [36,53,54]. Hoang, Brown [20] used a second-order three-dimensional structure of PA without the SB dimension in a World Cultural Heritage setting, since they considered the social component was more a reflection of residents’ attachment to the community instead of to the heritage site’s physical environment. This study examined local residents’ PA to the city or town they lived instead of the tourist attraction itself, it included the social component and provided empirical evidence for the reliability and validity of this PA measurement structure, which accurately reflected a WHS’s local residents’ cognitive, functional, emotional and social bonds with the place they live. Our results show PAF has the highest predictive power, followed by PD and SB, and PI has the lowest predictive power. This order is different from Ramkissoon, Smith [15] in the ranking of PI which comes in the second, and different from Hesari, Peysokhan [36] and Shaykh-Baygloo [54] in the position of the SB constituent which ranks first and last, respectively.

The results of the SEM confirm that residents’ PA positively influence their PP of heritage tourism of the Grand Canal in both the city and the towns. Significant differences are identified between this relationship in the city and town area along the canal, where PA had significantly greater effect on the town residents’ PP of the heritage tourism than that on the city residents. Few researches had directly studied the effect of residents’ PA on their PP. Some early studies investigated how community attachment influence perceptions of tourism impact but reached different conclusions. For instance, Um and Crompton [92] found that more community-attached residents were prone to have less PP of tourism impacts, while McCool and Martin [93] concluded that no clear connection exist between the two. Jurowski, Uysal [47] decomposed the concept of community attachment and discovered that more attached residents appeared to hold more PP on economic and social impacts but more NP on environmental impacts [49,50], while Gursoy, Jurowski [48] identified no significant relationship between community attachment and perceived cost and benefits. As the multidimensional concept of PA develops, recent studies of Stylidis [63] investigated the effect of PA on residents’ tourism perceptions and did not confirm a positive relationship, but his results may be interfered by the simultaneous test of place perception. Vong [19] confirmed a positive relationship between young students’ PP of heritage tourism and their PA but the results may be biased due to the specific age group and small sample size. This research firstly provides empirical evidence for that the more the residents attached to the place they live, the more positive economic, social and cultural benefits they perceive in linear WHS settings.

The article "City vs. Town residents’ place attachment, perceptions and support for tourism development in a linear World Cultural Heritage Site" was published in 2021. Journal: PLoS One.

Residents’ PA negatively impacts their NP in the town area but does not have statistical significance to those in the city area, and significant differences are revealed between these impacts. Town residents with greater PA are less likely to have negative economic, social and environmental perceptions towards tourism development while city residents’ PA have nearly no impact on their NP. There are few studies specifically include the relationship between residents’ PA and their NP, only community attachment was found to have significantly or non-significantly negative effect on residents’ NP in rural or urban heritage settings [50,66].

The findings show significant effects of residents’ PP on their ST, which is also seen in many former studies [58,61,67]. This effect was larger in the town area than that in the city area, which means PP of town residents evoke more supportive attitude for heritage tourism development than that of city residents within the same section of the canal, but no statistically significant differences are identified between the two effects. This result is different from Rasoolimanesh, Ringle [22] which discovered the effect size was significantly larger in the urban context than in the rural context. The city of Yangzhou’s tourism has been developing for many years, which was much earlier than the Grand Canal’s inscription on the World Cultural Heritage list, and local residents are more used to the benefits brought by tourism development, but the tourism development in those towns and villages started just after the inscription and local residents’ perceptions may generate stronger impact on their supportive attitudes.

The article "City vs. Town residents’ place attachment, perceptions and support for tourism development in a linear World Cultural Heritage Site" was published in 2021. Journal: PLoS One.

Town residents’ NP have significantly negative impacts on their ST while city residents’ NP have no statistically significant influence on their supports, and their differences are non-significant. This result supports previous studies which found that residents with NP were less supportive of tourism development in rural/town communities [22,59], but do not cohere with the findings in the urban setting which identified more supportive attitude of local residents who held NP [22]. One possible reason is that although Yangzhou downtown residents had recognized the negative economic, sociocultural and environmental influence of heritage tourism upon local communities, they have been experiencing the benefits brought by tourism for the past decades. When the positive impacts outweigh part of the negative impacts and local residents are more used and receptive to tourism development, residents’ NP contribute little to their supportive attitudes.

City residents’ PA to Yangzhou city has direct effect on their ST of the Grand Canal Yangzhou Section as well as indirect effect through their PP, which means partial mediation exists in these relationships. However, although within the same section, town residents’ PA has little direct effect on their ST, and the effect of PA on ST are fully mediated by their PP and NP. The overall results show that local residents’ PA works differently on their ST between city and town areas, and the possible reasons are that the cities usually have more tourism than the towns and the city residents are better educated than the town residents. City residents are generally more understanding and accustomed to tourism development due to their richer life experiences and higher education level, so their PA could directly lead to their ST as well as through PP. However, town residents are relatively more sensitive and critical of tourism development since those projects are usually new to them, and their PA would first influence their PP and NP of tourism development and then affect their attitude. Therefore, the findings of this study should be consistent in most cities and towns.

Theoretical contributions of this study include, first utilizing the four-dimension PA to measure a WHS residents’ bonds to the city or town they live, and test how this attachment affect their responses of tourism development; and second, comparing these effects among city and town residents within the same section along the same linear WHS site. Practical implications are that since urban residents’ attachment to the city itself can directly contribute to their tourism support, it is more important for the city government along with destination marketing organizations (DMOs) to improve the quality and attractiveness of the city as a whole as well as enhance the economic, sociocultural and environmental benefits of the Grand Canal heritage tourism. However, in order to increase town residents’ support towards heritage tourism, DMOs should play a leading role and focus more on increasing the positive impacts and reducing the negative impacts of heritage development projects so that residents can get better perceptions, such as creating better surrounding landscapes for those historic sites and providing high-quality public spaces and facilities nearby, publicizing the local history and culture of the Grand Canal, reducing the interference of tourism development on local residents’ lives, and minimizing the damage of tourism facility construction to the integrity of local villages and towns.

The article "City vs. Town residents’ place attachment, perceptions and support for tourism development in a linear World Cultural Heritage Site" was published in 2021. Journal: PLoS One.

## 6. Conclusions

This research utilized the concept of place attachment for understanding the bonding between local residents and their living place, and studied how it affects residents’ perceptions and support for tourism development. The findings assert that there is a positive meaningful relationship between place attachment and support for heritage development, and this relationship of city residents is direct and partially though positive perceptions while that of town residents is indirect and fully though residents’ positive and negative perceptions.

This research has some limitations which should be addressed in the future. First, group analyses based upon sociodemographic characteristics were not conducted. Since local residents have different characteristics, it will be interesting to test whether people’s gender, age, educational background, length of residence etc. moderate the model besides the city-town difference. Second, other than residents’ perceptions and support of tourism, their participatory behavior or behavioral intention are also important cornerstone of sustainable tourism development, which were not included in the study. The relationship between place attachment and community participation should be examined with the potential mediators and moderators adding to Hesari, Moosavy [53]’s model. Third, this study was conducted in Yangzhou Section of the Grand Canal, although it is one of the most ancient and influential section along the whole route, future research on the other typical sections should be carried out to obtain a panoramic view of local residents’ place attachment and tourism responses to a linear World Heritage and horizontal & vertical comparative analyses should be conducted. Bringing residents’ diversified attitudes and responses, the tourism development of a linear heritage site can be more targeted and sustainable.

The article "City vs. Town residents’ place attachment, perceptions and support for tourism development in a linear World Cultural Heritage Site" was published in 2021. Journal: PLoS One.

## Supporting information

S1 Dataset (XLSX)
